The article "Influence of Rib Cage on Static Characteristics of Scoliotic Spine" was published in 2020. Journal: Appl Bionics Biomech.

# Influence of Rib Cage on Static Characteristics of Scoliotic Spine

**DOI:** 10.1155/2020/8858686

**Published:** 2020-10-19

**Authors:** Liying Lin, Shaowei Jia, Hufei Yang, Ye Li, Shunxin Zhang, Jie Fan, Li Han

**Affiliations:** ^1^School of Medical Imaging, Tianjin Medical University, Tianjin 300203, China; ^2^Key Laboratory for Biomechanics and Mechanobiology of Ministry of Education, School of Biological Science and Medical Engineering, Beihang University, Beijing 100083, China; ^3^School of Mechanical Engineering, Hebei University of Technology, Tianjin 300130, China; ^4^Department of Orthopedics, Peking Union Medical College Hospital, PUMC&CAMS, Beijing, China; ^5^Department of Radiology, Tianjin Medical University General Hospital, Tianjin, China

## Abstract

**Background:**

Scoliosis is a three-dimensional (3D) deformity of the spine, which affects the patient's appearance and may lead to abnormal heart and lung function. The rib cage is a structure composed of ribs, sternum, and costal cartilage, which plays a vital role in stabilising the thoracolumbar spine. This study investigates the influence of the rib cage on the static characteristics of the scoliotic spine.

**Methods:**

Two types of 3D finite element (FE) models with or without rib cage (from T1 to S) were established and analysed based on computed tomography (CT) images, to determine the effects of the rib cage on the static characteristics of the scoliotic spine. The FE software, ABAQUS, was used to analyse the static behaviours of scoliotic spine models under a range of loading conditions, including left side bending, right side bending, front tilt, rear supine, and vertical compression. The changes in the von Mises stress (VMS) within the intervertebral discs of spine models with or without rib cage were studied and compared.

**Results:**

After including the rib cage, the maximum VMS at the stress concentrations of the normal and scoliotic spine effectively reduced. The VMS in normal intervertebral discs was gentler than that of scoliotic ones. However, the scoliotic spine was more likely to produce large stress concentration in the intervertebral discs of scoliotic segments.

**Conclusions:**

Under the common postures, intervertebral discs of scoliotic segments are more susceptible to generate stress concentrations compared with the normal spine. The rib cage could effectively keep the intervertebral discs of scoliotic segments from further injuries. These results are of great significance for the prevention and treatment of the scoliotic spine.

## 1. Introduction

Scoliosis is a deformity of the spine with lateral curvature in the coronal plane. This deformity can lead to anatomical changes in the structure of the rib cage, which could, in turn, cause changes in the mechanical properties of the spine. The deformity is a biomechanical process, which is part of a vicious cycle, especially under external loads [1]. Severe scoliosis can lead to a “razor-back” appearance, which not only affects the patient's physical appearance but can also lead to abnormal heart and lung function [2–4]. The rib cage is composed of the sternum, ribs, costal cartilage, and rib joints, which is an important anatomical structure of the thoracic spine. It can enhance respiration, protect the organs in the thoracic cavity, and provide stability and share the load of the spine [5–7].

To investigate the role of the rib cage in the stability of the spine, scholars have used various methods to study the relationship between them. Previous studies have studied the biomechanics of the rib cage and proved that the rib cage contributes to mechanical stability to the spine [8–11]. Watkins et al. used experiments on cadaver specimens to study the effect of the rib cage on the stability of the normal spine under external load [12]. Gignac et al. used the finite element (FE) method to study the best loading patterns required to correct both the spine and the rib cage scoliotic deformities [13]. Mannen used cadaver specimens to study the changes in the mechanical properties of the rib cage of a normal spine [14]. Previous studies have lacked the effect of the thoracic cage on the spine due to the absence of cadaver samples, but finite element analysis of the spine can compensate for this.

In this study, four FE models, including normal spine without rib cage (NS1), normal spine with normal rib cage (NS2), scoliotic spine without rib cage (SS1), and scoliotic spine with deformed rib cage (SS2), were selected. Under the conventional postures, such as left side bending, right side bending, front tilt, rear supine, and vertical compression, the effects of the rib cage on the static characteristics of the scoliotic spine were studied by comparing the von Mises stress (VMS) changes within the intervertebral disc of the scoliotic spine. The normal spine was used as the control group to investigate the protective effect of the rib cage on the intervertebral disc of the scoliotic spine. This study provides a basis for mechanical analysis of thoracoplasty and prevention of scoliosis.

## 2. Materials and Methods

### 2.1. Establishment of the Finite Element Model

In this study, a scoliotic spine and a normal spine were selected as the study subjects. Written informed consent was obtained from all participants of the study. A computed tomography (CT) scanner (64-slice spiral CT, Siemens, Germany) was used at the Beijing Union Hospital for imaging of the thoracolumbar area of the scoliotic spine and the normal spine. The scanning parameters were a tube voltage of 120 kilovolts (kV), tube current of 211.20 milliamperes (mAs), interlayer spacing of 0.625 millimetres (mm), and matrix of 512 × 512 pixels. Each scan has a total of 867 transaxial slices obtained in Digital Imaging and Communications in Medicine (DICOM) format.

The software Mimics 16.0 (Materialise NV, Belgium) was used to construct a basic 3D model of the vertebrae and the rib cage. A smooth 3D model of the vertebrae and rib cage was obtained using Geomagic Studio (Geomagic Inc., USA) software. By performing Boolean calculation, three parts were created, including (1) structure of vertebrae composed of cortical bone, cancellous bone, and the posterior part of the vertebrae; (2) structure of the intervertebral disc composed of the annulus fibrosus, nucleus pulposus (which takes up one-third of the discs and is located at the posterior end), and upper and lower endplates; and (3) structure of the rib cage composed of the sternum, ribs, costal cartilage, and rib joints. Four FE models, including NS1, NS2, SS1, and SS2, were developed in the FE software, Abaqus 6.14 (Dassault SIMULIA Inc., France). The upper 12 vertebrae are the thoracic vertebrae (T1-T12, from top to bottom), the next 5 are lumbar vertebrae (L1~L5, from top to bottom), and the last one is the sacrum, S; all four FE models are shown in Figure 1.

Figure 1 shows that the normal spine was symmetrical on the left and right sides, while the vertebrae of the scoliotic spine deviated from the midline. There was a right side curvature of the Cobb angle of about 60° at T5~T6 (first side convex) and a left side curvature of the Cobb angle of about 30° at T11~T12 (second side convex).

The four sets of geometric models, as shown in Figure 1, were meshed in 3-Matic in the software Mimics 16.0. Each edge of the element size was set to about 1 mm, and the mesh element type used in this research model was C3D4 element. The quality of the mesh was up to standard qualified in the software testing. The FE models of vertebral bodies and intervertebral discs are shown in Figure 2.

The mesh models were assigned the specific material properties, as shown in Table 1 [15–18].

A ligament simulated by a linear tension spring was added between the vertebrae. According to the human body anatomy, spring was used to simulate human ligament and was added to the corresponding position in this study. The stiffness formula of the spring is as shown in

(1) $$\begin{array}{c} k=\frac{E\cdot A}{L}, \end{array}$$

where *k* is the stiffness of the spring, *E* is the elastic modulus, *A* is the cross-sectional area, and *L* is the average length. The material properties of the ligaments are based on published data, as shown in Table 2 [11, 19]. The supraspinous ligament, interspinous ligaments, anterior longitudinal ligament, posterior longitudinal ligament, intertransverse ligaments, and ligamentum flavum in the thoracolumbar segment were stimulated. The ligaments between the ribs were not considered due to lack of published data.

At present, the primary means of validating the existing models of the spine is to compare them with the cadaver specimen, under the same experiment boundary conditions [20]. To prove the reliability of the proposed FE model, we only chose those parts of the lumbar vertebra model that were previously studied in the literature. The model proposed in this study was validated under physiological loading modes: (1) compression, (2) anterior and posterior shear, and (3) the predicted responses were compared against results by Berkson et al. [21] and Xiang et al. [22] under similar boundary and loading configurations. The predicted displacement values at the centre of the superior vertebral body (under compression and shear loading) were compared to the aforementioned *in vitro* experimental results.

### 2.2. Static Analysis

#### 2.2.1. Selecting Poses for Static Analysis

Given the complexity of human body movement during daily life and travel, the spine movements were simplified to postures such as left side bending, right side bending, front tilt, rear supine, and vertical compression. The static analysis of simple postures of the spine structure can reflect the static characteristics of the complex motion of the human body. Therefore, static analyses of four spine models, including NS1, NS2, SS1, and SS2 were performed in various simple poses. The VMS changes in the intervertebral disc were compared before and after adding the rib cage at each posture.

#### 2.2.2. Adding Boundary Conditions and Loads

The effect of the rib cage on the intervertebral disc of the scoliotic spine in common postures was analysed. The vertebrae of the spine are connected through the intervertebral disc. The upper and lower endplates of the intervertebral disc connect the annulus fibrosus and the nucleus pulposus. According to the anatomical properties of the spine tissue and the common postures in daily life, the tie constraints were used to fix all the existing contact surfaces. Also, it was necessary to constrain the six degrees of freedom on both sides of the sacrum of the four spine models. In order to simulate a simple posture of the human body, point-to-surface coupling was created on the right, left, back, front, and top of the first thoracic vertebra (T1), respectively. An external load was applied to the coupling point, and a point mass of 10.5 kilograms (kg) was added to the upper surface of T1 of the four models to simulate the influence of the mass of the head, neck, and upper limbs on the spine model to improve the analysis [3, 23]. The same loads and boundary conditions were added to the four spine models in the same posture, as listed in Table 3.

## 3. Results

### 3.1. FE Model Validation

A comparison of the FE model and experimental results is shown in Figure 3. Under an axial pressure of 400 Newton (N) and the anterior and posterior shear force of 86 N, the calculated displacements of the centre of the L1-L4 vertebral surface in the vertical direction fall within the range of the aforementioned experimental data. These results align well with the experimental findings of Berkson et al. [21]. Moreover, the vertical displacements are close to the FE data of Xiang et al. [22]. Therefore, the scoliosis model established in the study is validation and reliable.

### 3.2. Results of Static Analysis

All the intervertebral discs of the thoracic and lumbar vertebrae T1~S were selected as the research object. The maximum VMS on the intervertebral disc was obtained under various simple postures of the same load. The change of the equivalent stress of the intervertebral disc in the same posture before and after adding the rib cage was studied.

#### 3.2.1. Static Analysis Results of Left and Right Side Bending

Under the same external load, the left and right side bending of the spines was simulated, and the equivalent stresses on the intervertebral discs of four FE models were studied. The VMS distribution cloud diagrams are shown in Figures 4 and 5. The maximum VMS on the intervertebral disc of the four spine models was measured and plotted as the stress distribution map of the intervertebral disc of the whole spine, as shown in Figures 6 and 7.

As shown in Figures 4–7, under the same loading conditions, the VMS of the intervertebral disc of the normal spine T1~S showed an increasing trend, and the overall VMS was smaller and more stable than that of the scoliotic spine. The VMS of the intervertebral disc of the scoliotic spine T1~S showed an increasing trend, and the overall VMS was larger than the normal spine. There were mutations near the scoliotic segments T4, T8, and T12, presenting three distinct peaks. In the normal spine with the rib cage, the VMS of the intervertebral disc of T1~T12 was slightly reduced, and the VMS of the intervertebral disc of L1~L5 was slightly increased. In the scoliotic spine with the deformed rib cage, the VMS of the intervertebral disc of T1~T12 was significantly reduced, and the VMS of the intervertebral disc of L1~L5 was significantly increased.

#### 3.2.2. Static Analysis Results of Front Tilt and Rear Supine

Under the same external load, the front tilt and rear supine were simulated, and the equivalent stresses on the intervertebral disc of four models were studied. The VMS distribution cloud diagrams are shown in Figures 8 and 9. The maximum VMS on the intervertebral disc was measured and plotted as the stress distribution map, as shown in Figures 10 and 11.

As shown in Figures 8–11, under the same loading conditions, the VMS of the intervertebral disc of the normal spine T1~S showed an increasing trend, and the overall VMS was smaller and more stable than that of the scoliotic spine. The VMS of the intervertebral disc of the scoliotic spine T1~S showed a normal distribution trend, and the overall VMS was larger than the normal spine. There was a peak near the scoliotic segment T8, gradually decreasing on both sides. In the normal spine with the rib cage, the VMS of the intervertebral disc of T1~T8 was significantly reduced, and the VMS of the intervertebral disc of L1~L5 was slightly increased. In the scoliotic spine with the deformed rib cage, the VMS of the intervertebral disc of T1~T12 was significantly reduced, and the VMS of the intervertebral disc of L1~L5 was significantly increased.

#### 3.2.3. Static Analysis Results of Vertical Compression

Under the same external load conditions, the vertical compression was simulated, and the equivalent stress on the intervertebral disc of four models was studied. The VMS distribution cloud diagram is shown in Figure 12. The maximum VMS on the intervertebral disc was measured and plotted as the stress distribution map, as shown in Figure 13.

As shown in Figures 11 and 12, under the same loading conditions, the VMS of intervertebral discs of the normal spine T1~S showed a decreasing trend, and the overall VMS was smaller and more stable than that of the scoliotic spine. The VMS of intervertebral discs of the scoliotic spine T1~S showed a trend of M-type distribution, and the overall VMS was large larger than the normal spine. There were two peaks near the scoliotic segments T4 and T10, gradually decreasing on both sides. In the normal spine with the rib cage, the VMS of the intervertebral disc of T1~T8 was significantly reduced, and the VMS of the intervertebral disc of L1~L5 did not change significantly. In the scoliotic spine with the deformed rib cage, the VMS of the intervertebral disc of T1~T12 was significantly reduced. The scoliotic segments T4 and T10 had the most significant reductions, and the VMS of the intervertebral disc of L1~L5 did not change significantly.

## 4. Discussion

Scoliosis is a 3D deformity of the spine, which experiences asymmetrical loading. Few studies investigated cadaveric specimens of the scoliotic spine due to the lack of cadaver specimens, so FEM and FE analyses have been a useful tool to simulate the cadaver specimens. In this study, four FE models were established, and static behaviours of scoliotic spine models (with or without rib cage) were assessed under the conventional postures.

Compared with the vertebrae, the intervertebral disc is more susceptible to deformation and damage under external load [24]. In this study, we compared the VMS of the intervertebral discs on T1~S of the thoracolumbar vertebrae of the scoliotic and normal spine model with and without rib cage. After the rib cage was added to the normal spine, the VMS of the intervertebral disc of the thoracic vertebrae generally reduced. The results imply that the rib cage can increase the stability of the thoracic spine, confirming the conclusions of the previous studies [12, 14]. After the addition of rib cage, the stress of intervertebral discs of the normal spine reduced more evenly, while the stress of the scoliotic spine was concentrated on the scoliosis segments, and the reductions of the stress after the addition of rib cage were also concentrated with the scoliosis segments. The result may be explained by the characteristics of the spinal structure of the scoliotic spine.

The research presented in this manuscript has laid a foundation for the further mechanical studies of idiopathic scoliosis. The study has several limitations. The material properties of the models are based on generally accepted data. However, the bone material properties may be different with different individuals, genders, ages, and pathological spines. Therefore, the material properties of specific spine will be needed to be improved further. Only five postures were studied in this study, and each posture was simulated with one force. In reality, the posture of the human body is very complicated and requires multiple forces to simulate. Also, muscle tissue near the thorax, spine, and pelvis affect the force and dynamics of the spine. In subsequent studies, these components need to be included to bring the model and findings closer to reality for clinical research.

## 5. Conclusions

Intervertebral discs of scoliotic segments generate stress concentrations more commonly compared with normal spine under common postures. The rib cage can protect the intervertebral discs of scoliotic segments. The rib cage mainly protects different segments in different postures. These results are of great significance for the prevention and treatment of the scoliotic spine. This study provides useful references for the treatments and protection of scoliosis patients and the development of scoliosis medical devices and related products.

## Figures and Tables

**Figure 1:** Four finite element models are shown: (a) normal spine without rib cage (NS1); (b) normal spine with normal rib cage (NS2); (c) scoliotic spine without rib cage (SS1); (d) scoliotic spine with deformed rib cage (SS2).

**Figure 2:** The mesh of vertebral bodies and intervertebral discs are shown: (a) cortical bone; (b) cancellous bone; (c) vertebra; (d) annulus fibrosus; (e) nucleus pulposus; (f) upper and lower endplates; (g) spinal segment.

**Figure 3:** Comparison of FE analysis and experimental results: (a) lumbar vertebral deformation under an axial pressure of 400 N; (b) lumbar vertebral deformation under an anterior shear force of 86 N; (c) lumbar vertebral deformation under a posterior shear force of 86 N.

**Figure 4:** von Mises stress distribution of discs in four spinal models with left curvature: (a) normal spine without rib cage (NS1); (b) normal spine with normal rib cage (NS2); (c) scoliotic spine without rib cage (SS1); (d) scoliotic spine with deformed rib cage (SS2).

**Figure 5:** Stress distribution of discs in four spinal models with left curvature: (a) stress distribution of normal spinal intervertebral disc; (b) stress distribution of scoliotic spinal intervertebral disc. NS1, NS2, SS1, and SS2 need to be defined here.

**Figure 6:** von Mises stress distribution of discs in four spinal models with right curvature: (a) normal spine without rib cage (NS1); (b) normal spine with normal rib cage (NS2); (c) scoliotic spine without rib cage (SS1); (d) scoliotic spine with deformed rib cage (SS2).

**Figure 7:** Stress distribution of discs in four spinal models with right curvature: (a) stress distribution of normal spinal intervertebral discs; (b) stress distribution of scoliotic spinal intervertebral discs. NS1, NS2, SS1, and SS2 need to be defined here.

**Figure 8:** von Mises stress distribution of disc in four spinal models with anterior tilt: (a) normal spine without rib cage (NS1); (b) normal spine with normal rib cage (NS2); (c) scoliotic spine without rib cage (SS1); (d) scoliotic spine with deformed rib cage (SS2).

**Figure 9:** Stress distribution of disc in four spinal models with anterior tilt: (a) stress distribution of normal spinal intervertebral discs; (b) stress distribution of scoliotic spinal intervertebral discs. NS1, NS2, SS1, and SS2 need to be defined here.

**Figure 10:** von Mises stress distribution of disc in four spinal models with posterior supine: (a) normal spine without rib cage (NS1); (b) normal spine with normal rib cage (NS2); (c) scoliotic spine without rib cage (SS1); (d) scoliotic spine with deformed rib cage (SS2).

**Figure 11:** Stress distribution of disc in four spinal models with posterior supine: (a) stress distribution of normal spinal intervertebral discs; (b) stress distribution of scoliotic spinal intervertebral discs. NS1, NS2, SS1, and SS2 need to be defined here.

**Figure 12:** von Mises stress distribution of disc in four spinal models under vertical compression: (a) normal spine without rib cage (NS1); (b) normal spine with normal rib cage (NS2); (c) scoliotic spine without rib cage (SS1); (d) scoliotic spine with deformed rib cage (SS2).

**Figure 13:** Stress distribution of disc in four spinal models under vertical compression: (a) stress distribution of normal spinal intervertebral discs; (b) stress distribution of scoliotic spinal intervertebral discs. NS1, NS2, SS1, and SS2 need to be defined here.

**Table 1:** The material attributes of various spine structures.

Structure	Unit type	*E* (MPa)	*ν*	*ρ* (T·mm^−3^)
Cortical bone	Tetrahedral unit	12000	0.30	1.7*E*-9
Cancellous bone	Tetrahedral unit	150	0.30	1.1*E*-9
Posterior part	Tetrahedral unit	3500	0.30	1.4*E*-9
End plate	Tetrahedral unit	100	0.40	1.2*E*-9
Annulus fibrosus	Tetrahedral unit	4	0.45	1.05*E*-9
Nucleus pulposus	Tetrahedral unit	1	0.499	1.02*E*-9
Ribs	Tetrahedral unit	5000	0.30	2.0*E*-9
Intercostal cartilage	Tetrahedral unit	480	0.40	2.0*E*-9
Sternal	Tetrahedral unit	10000	0.30	2.0*E*-9

*E*: elastic modulus; *ν*: Poisson's ratio; *ρ*: density.

**Table 2:** The structural attributes of the major ligaments in the thoracolumbar sacral spine.

Main ligament	*E* (MPa)	*k*	*L* (mm)	*A* (mm^2^)
Anterior longitudinal ligament	7.8	8.74	20	22.4
Posterior longitudinal ligament	10	5.83	12	7.0
Ligamentum flavum	17	15.38	15	14.1
Intertransverse ligaments	10	0.19	32	0.6
Interspinous ligaments	10	10.85	13	14.1
Supraspinous ligament	8.0	2.39	22	10.5

**Table 3:** The external load addition in four spinal models [10].

The posture of the spine model	The load of the four spinal models
Left side bending	Add 100 N force from right to left on T1
Right side bending	Add 100 N force from left to right on T1
Front tilt	Add 100 N force from the back to the front on T1
Rear supine	Add 100 N force from the front to the back on T1
Vertical compression	Add 100 N force from top to bottom on T1

## Data Availability

The datasets used during the current study are available from the corresponding author on reasonable request.
